# Efficient Detection Method of Pig-Posture Behavior Based on Multiple Attention Mechanism

**DOI:** 10.1155/2022/1759542

**Published:** 2022-07-16

**Authors:** Li Huang, Lijia Xu, Yuchao Wang, Yingqi Peng, Zhiyong Zou, Peng Huang

**Affiliations:** College of Mechanical and Electrical Engineering, Sichuan Agriculture University, Ya'an 625014, China

## Abstract

Due to the low detection precision and poor robustness, the traditional pig-posture and behavior detection method is difficult to apply in the complex pig captivity environment. In this regard, we designed the HE-Yolo (High-effect Yolo) model, which improves the Darknet-53 feature extraction network and integrates DAM (Dual attention mechanism) of channel attention mechanism and space attention mechanism, to recognize the posture behaviors of the enclosure pigs in real-time. First, the pig data set is clustered and optimized by the K-means algorithm to obtain a new anchor frame size. Second, the DSC (Depthwise separable convolution) and h-switch activation function are innovatively introduced into the Darknet-53 feature extraction network, and the C-Res (Contrary residual structure) unit is designed to build Darknet-A feature extraction network, so as to avoid network gradient explosion and ensure the integrity of feature information. Subsequently, DAM integrating the spatial attention mechanism and the channel attention mechanism is established, and it is further combined with the Incep-abate module to form DAB (Dual attention block), and HE-Yolo is finally built by Darknet-A and DAB. A total of 2912 images of 46 enclosure pigs are divided into the training set, the verification set, and the test set according to the ratio of 14 : 3:3, and the recognition performance of HE-Yolo is verified according to the parameters of the precision *P*, the recall *R*, the AP (i.e., the area of P-R curve) and the MAP (i.e., the average value of AP). The experiment results show that the AP values of HE-Yolo reach 99.25%, 98.41%, 94.43%, and 97.63%, respectively, in the recognition of four pig-posture behaviors of standing, sitting, prone and sidling of the test set. Compared with other models such as Yolo v3, SSD, and faster R–CNN, the mAP value of HE-Yolo is increased by 5.61%, 4.65%, and 0.57%, respectively, and the single-frame recognition time of HE-Yolo is only 0.045 s. In the recognition of images with foreign body occlusion and pig adhesion, the mAP values of HE-Yolo are increased by 4.04%, 4.94%, and 1.76%, respectively, while compared with other models. Under different lighting conditions, the mAP value of HE-Yolo is also higher than that of other models. The experimental results show that HE-Yolo can recognize the pig-posture behaviors with high precision, and it shows good generalization ability and luminance robustness, which provides technical support for the recognition of pig-posture behaviors and real-time monitoring of physiological health of the enclosure pigs.

## 1. Introduction 

China is the world's largest producer of pigs and a major consumer of pork. According to statistics, 337.42 million pigs were sold in the first half of 2021, a year-on-year increase of 34.2% compared with 2020. The 2019 China statistical yearbook shows that China's per capita meat consumption is 26.9 kg/person, and the consumption proportion of pork in meat products is as high as 60%. This shows that pig breeding is the most important industry in China's animal husbandry, which is of great significance to national life, stabilizing prices, ensuring the smooth operation of the economy, and stabilizing the overall social situation. Most of China's pig breeding industry is still dominated by periodic manual supervision, with high labor intensity, low work efficiency, poor timeliness, and easy to make mistakes. It is imperative to use the information and intelligent technical means to detect the behavior and posture of pigs in real time.

At present, many scholars applied CNN (convolutional neural networks) to recognize multi-category targets [1–5] in different fields. In pig-posture behavior recognition, Gao et al. [6] used a 3D convolutional network to recognize the aggressive pig behaviors, but some interference factors such as pig adhesion, different lightings, and complex behaviors resulted in a weak generalization ability of CNN. Zhou et al. [7] designed a pig face detection method with an attention mechanism [8–10] combined with a feature pyramid structure, which made the network more focused on the effective information area of the images, but the gradient dispersion appeared with the deepening of the number of the network layers. Yang et al. [11] used CNN to recognize the individual pig-drinking behaviors, but the method showed the complex calculation of feature selection and relied on high hardware. Zheng et al. [12] used the faster R–CNN to recognize the standing, lying, and the other behaviors of sows, but the recognition results of different scales of targets were quite different. The R–CNN series networks designed in the literature [13–15] generated sample feature maps through convolution processing of input images, and then classify them. The experimental results showed that these networks were not very effective to recognize the multi-scale small targets. The Yolo series networks designed in the literature [16–18] converted the positioning of the target frames into a regression problem, which showed high recognition accuracy and short recognition time. Among them, the Darknet-53 feature extraction network of Yolo v3 was characterized by a large calculation, unstable gradient, and incomplete feature information extraction, and the feature information of each region of the feature map was given the same weight. In fact, the contribution degrees of feature information of some areas such as pig-limbs, pig-abdomen, and pig-trunk were far greater than that of pig-head, pig-feces and pig-pigsty. Therefore, it is considered to introduce DAM (i.e., dual attention mechanism) to focus more on the target areas.

To realize the real-time recognition of the pig-posture behaviors in the enclosure environment, a DSC (i.e., depthwise separable convolution) structure and h-switch activation function are introduced into the Darknet-53, and C-Res (i.e., contrary residual structure) unit is designed. Further, DAM is combined with Incep-abate to form the DAB (i.e., dual attention block), so as to reduce the computational complexity and the hardware cost of the network, and further reduce its false recognition rate. The rest remainder of this study is organized as follows. In Section 2, the pig mages are acquired and preprocessed, and the building process of HE-Yolo model is described. In Section 3, Experiments are conducted using the pig mages with four pig-posture behaviors in an enclosure environment, and the results are analyzed and discussed. Finally, the conclusions of this study are drawn in Section 4.

The detection method proposed in this paper can be used to infer the movement state of captive pigs. Based on this technology, the active state of pigs in a fixed time can be judged, and the judgment index of pig activity degree can be generated, which provides effective help for the follow-up behavior research and physiological condition analysis of pigs.

## 2. Materials and Methods

### 2.1. Experimental Image Preparation

#### 2.1.1. Subsection

The pig images are acquired from a pig farm in Guang'an city of Sichuan province (10 : 00–14 : 00 on August 14th, 2021, with cloudy weather) and another pig farm in Leshan city of Sichuan Province (10 : 00–14 : 00 on August 14th, 2021, with sunny weather). Canon EOS580D anti-shake camera is 0.5∼2.0 m away from the pig-body to take photos of pig-trunk of different scales. The sizes of the two pig farms are 10 m × 5 m × 0.7 m and 8 m × 6 m × 0.8 m, with 2∼10 pigs in each column. A total of 46 pigs in three columns in a nursery period of 24∼54 days and a fattening period of more than 70 days are selected as the study objects.

The postural behaviors of pigs vary greatly, which are usually divided into four categories: standing, sitting, prone, and sidling. A total of 30 segments of video data of pigs are manually screened, with each segment of 10∼100 s, and 728 images with a resolution of 1920 × 1080 are obtained by frame-by-frame processing. To expand the number of images and improve the universality of the network, we perform −10° flip, +10° flip, mirror flip, and random luminance adjustment on the images to expand the data set (shown in Figure 1). After expansion, a data set of 2912 images is obtained.

#### 2.1.2. Devising the Image Data

Take the pig-limb, the pig-abdomen, and the pig-trunk as the dividing points and do not mark the pig images in which any two of three parts do not appear within the marking range. The open-source tool labeling [19] is used to label the images with four pig-posture behaviors, namely “standing”, “sitting”, “prone” and “sidling”. According to the general division strategy [20], the labeled extended dataset is divided into the training set of 2040, the validation set of 436, and the test set of 436 according to the ratio of 14 : 3:3, and with the resolution of 1920 × 1080 × 3. The images are further scaled and converted into the network with a resolution of 416 × 416. After labeling all images, the coordinates of the marked parts are transformed to obtain the coordinates of the scaled corresponding parts, as shown in Figure 2.

### 2.2. Building HE-Yolo

The Yolo series network is mainly composed of a pooling layer and convolution layer, and the resolution of the input image is 416 × 416. The input image is processed by a series of 3 × 3 depthwise convolution and 1 × 1 pointwise convolution, pooling, and up-sampling operations to output the feature map. Darknet-53 consists of 1 × 1 pointwise convolution and 3 × 3 depthwise convolution layers, and the batch normalization layer and Leaky ReLU concatenated after each convolutional layer are to prevent overfitting. The convolutional layer, batch normalization layer, and Leaky ReLU activation function together form the basic convolution unit DBL of Darknet-53, with a total of 53 DBL units. To predict the multi-scale small targets, Yolo v3 uses anchor boxes of 9 sizes. According to the idea of a feature pyramid network, Yolo v3 designs 3 sizes of network outputs to predict the targets of different scales, and its multi-scale feature extraction module shows strong recognition ability. The multi-scale feature map has multiple recognition results for the same target, so Yolo v3 introduces nonmaximum suppression [21] to eliminate the redundant detection frames, thus each target has a unique detection frame, and each area in the input feature map is assigned to an equal weight. The pig-trunk, the pig-abdomen, the pig-limb, the pig-feces, and the pig-pen in the images have different contributions to recognize the pig-posture behaviors. The weights of the feature information of the pig-feces, the pig-pen, and the other interfering feature information should be reduced, and the weights of feature information of the g-trunk, the pig-abdomen, and the pig-limb should be strengthened to improve the recognition accuracy of the pig-posture behaviors.

#### 2.2.1. Darknet-A Network

The DSC [22] and the h-switch activation function are introduced into the Darknet-53, and the C-Res unit is designed to build the Darknet-A feature extraction network.

*(1) DBH Unit*. The four pig-posture behaviors of standing, sitting, prone and sidling are closely related. Considering that the large sizes of pigs make it difficult to classify the behaviors, DSC and h-switch activation functions are introduced into Yolo v3 to reconstruct the structure of DBL of Darknet-53, that is, to form the DPH unit, so as to improve the recognition ability of network and reduce the amount of calculation. The structure of the DPH unit is shown in Figure 3.

The DSC decomposes the ordinary convolution in DBL into 3 × 3 depthwise convolution and 1 × 1 pointwise convolution, as shown in Figure 3. Of which, 3 × 3 depthwise convolution used different filters to convolve different channels of the input feature map, and then the feature maps outputted by 3 × 3 depthwise convolution are further weighted and combined by 1 × 1 pointwise convolution. Assume that the input feature map has *M* channels, the output feature map has *N* channels, and the size of convolution kernel is *D*_*k*_ × *D*_*k*_ then the amount of calculation of the depthwise convolution and the standard convolution is compared as follows:

(1) $$\begin{array}{c} \frac{H\times W\times M\times D_{k}\times D_{k}+H\times W\times M\times N}{H\times W\times M\times N\times D_{k}\times D_{k}}=\frac{1}{N}+\frac{1}{D_{k}}, \end{array}$$

where *N* ≫ *D*_*k*_. When *D*_*k*_=3 , the parameter quantity of DSC is about 1/9 of the standard convolution, which means that the DSC can greatly reduce the amount of calculation of Darknet-53.

The Leakly Relu activation function is used in DPH, and its gradient value is zero when the input is negative. As a result, the corresponding parameters of the input feature map will not be updated, and the data expansion will become more significant with the deepening number of network layers, thus it affects the recognition result of Yolo v3. The above problem can be solved by replacing the Leakly Relu activation function with the h-switch activation function [23]. The *h*-switch activation function is as follows:

(2) $$\begin{array}{c} f\left(x\right)=x\frac{\text{Relu}6\left(x+3\right)}{6}, \end{array}$$

where Relu6 () is the Relu activation function, but its maximum output is limited to 6.

The curve of the h-switch activation function is shown in Figure 4. It can be seen from Figure 4 that when *x*⟶−*∞*, *f*(*x*)⟶0.That is, the change trend of the *h*-switch activation function is similar to that of the Leakly Relu function, but when *x* is near 0, the gradient of the *h*-switch function will not completely disappear, which ensures the integrity of the feature information of the pig behaviors, and the *h*-switch activation function also reduces the computation complexity of the network.

*(2) C-Res Unit*. In the training process of a network based on the stochastic gradient descent algorithm, with the deepening of the network layers, the error is easy to cause gradient dispersion and gradient explosion through multi-layer back propagation. Therefore, the C-Res unit is designed based on the residual structure of Resnet.

Assuming there is a convolutional neural network, the input feature map needs to undergo *N* times of feature extraction, and each feature extraction corresponds to a nonlinear transformation *Z*_*i*_. *Z*_*i*_ is a set of multiple functions, such as the depthwise separable convolution, the activation function, the down sampling or pooling, etc. So there is as follows:

(3) $$\begin{array}{c} y_{i}=Z_{i}\left(y_{i-1}\right), \end{array}$$

where *y*_*i*_ and *y*_*i*−1_ represent the feature maps outputted by the *i*th layer and the (*i*-1) th layer, respectively.

The C-Res unit is expressed as follows:

(4) $$\begin{array}{c} y_{i}=Z_{i}\left(y_{i-1}\right)+y_{i-1}. \end{array}$$

The structure of the C-Res unit is shown in Figure 5.

Compared with the ordinary residual structure, the C-Res unit first raises the input feature map to a higher dimension and extracts its features by 3 × 3 depth convolution, and further reduces the dimension of the features, so as to reduce the computational load of Darknet-A and avoid gradient explosion.

#### 2.2.2. DAB

*(1) The Spatial Attention Block*. Spatial attention mechanism (SAM) [24] can enhance the target features in the input feature map. SAM assigns different weights to the pixels in the input feature map, and simultaneously performs global max pooling and global average pooling on all features of different channels in the same position, and then obtains two feature maps, which are further concatenated in the channel dimension to gain the initial spatial attention feature map of *H* × *W* × 2. Subsequently, 7 × 7 × 1 convolutional layer is used to reduce the initial spatial attention feature map to one channel, and generate the spatial weight coefficients through the sigmoid activation function. Then the spatial weight coefficients are multiplied with the input feature map through the residual structure to obtain the output feature map of SAM. The structure of the SAM module is shown in Figure 6.

*(2) The Channel Attention Block*. Channel attention mechanism (CAM) [25] weights the features of all channels of the input feature map to strengthen the effective features and weaken the irrelevant information. Among them, the global average pooling is used to aggregate the feature information contained in each spatial channel [26, 27], and the input feature map of *H* × *W* × *C* is pooled by global average pooling to obtain two-dimensional compressed feature of 1 × 1 × *C*. Global average pooling extracts the features of all areas of the feature map with equal weight, while global max pooling only calculates the area with the largest feature response, so it can make up for the deficiency of global average pooling in extracting channel attention information in the effective feature region. The structure of CAM module is shown in Figure 7.

*(3) The Channel Attention Block*. SAM and CAM are connected in series to build a dual attention mechanism (DAM). First, SAM is used to model the feature elements of the input feature map, so as to obtain the positional relationship between the feature elements and filter the spatial information, and then connect them through the residual structure and multiply by space to obtain the spatial attention feature map. Then, CAM is introduced to model the correlation between the channels of the spatial attention feature map, so that the feature elements in each position of the spatial attention feature map can obtain the corresponding spatial information, and they are also connected by the residual structure and multiplied by space, that is, the output feature map of DAM can be obtained. The structure of DAM module is shown in Figure 8.

*M* and *M*_0_ represent the input and the output feature maps of the DAM module, respectively, and their dimensions ∈*R*^*H*×*W*×*C*^. *F*_*S*_ represents the spatial weight coefficients generated by SAM, and *F*_*C*_ represents the channel weight coefficients generated by CAM, *F*_*S*_, *F*_*C*_ ∈ (0,1). *M*_0_ is calculated as follows:

(5) $$\begin{array}{c} M_{0}=\left(1+F_{C}\left(\left(1+F_{S}\left(M\right)\right)\times M\right)\right)\times \left(1+F_{S}\left(M\right)\right)\times M. \end{array}$$

Based on the principle of thermodynamics, the output feature map *M*_0_ obtained by DAM is converted into a heat map, and the visualization results of the feature information of key areas such as the pig-trunk, the pig-abdomen, and the pig-limb are shown in Figure 9.

DAM increases the computational complexity of the network. Since the Inception-v4 [28] module builds deeper and wider residual connections, the Incep-abate module is combined with DAM to form DAB. The average pooling, the max pooling, the asymmetric convolution, and 1 × 1 and 3 × 3 convolution layers are stacked together by using a parallel structure, and then the feature maps of each branch are fused by concat to ensure the integrity of the output feature map. Among them, 1 × 1 convolution changes the number of the channel layers of the input feature map, and the pooling layer changes the dimension of the input feature map. The Incep-abate module is an asymmetric convolution structure, and *N* × *N* × *C* convolution is replaced with 1 × *N* × *C* convolution and *N* × 1 × *C* convolution to reduce the hardware cost and improve the computing efficiency. The structure of the Incep-abate module is shown in Figure 10.

#### 2.2.3. HE-Yolo

HE-Yolo (high effection-Yolo) is built by Darknet-A and DAB, as shown in Figure 11. Darknet-A (i.e., the dotted box 1 in Figure 11) is used to compress the calculation of the feature map to reduce the occupation of hardware resources and ensure that feature information is not distorted. DAB (i.e., the dotted box 2 in Figure 11) obtains the coefficient matrix of the effective features through the operations such as the global max pooling, the global average pooling, and the sigmoid activation function to filter the features of the input feature map. HE-Yolo constructs a feature pyramid to achieve multi-scale feature fusion and improves the context semantics of the feature map through the intersection of multi-layer feature information. At the same time, nonmaximum suppression is applied to remove the detection frames with large deviations, so that each target corresponds to a unique detection frame.

The anchor box size of Yolo v3 is obtained by clustering on the coco data set, which is different from the posture behavior size of pigs. Therefore, a new anchor box size is set to improve the training effect of HE-Yolo. The K-means algorithm is used to cluster and optimize the labeled images to obtain the anchor box sets of three sizes of the pig image data set, as listed in Table 1.

## 3. Results and Analysis

### 3.1. Experimental Environment

Intel (R) core (TM) i7-6700 server with 32 GB memory and equipped with windows 10 operating system. Pychram integrated development environment and TensorFlow open-source library for parallel computing on GPU. GPU is configured as Nvidia GeForce RTX 5000 and GPU memory is 16 GB. The parallel computing environment is CUDA 9.0, cuDNN v7.4.2 and the programming language is Python 3.6.0. There are 2040 images in the training set. The small batch gradient descent training method is adopted and the number of iterations is set to 100. The initial learning rate is set to 0.001 and the learning rate is adjusted by the epoch-decay strategy. When the Intersection over Union (IoU) of the detection frame is greater than the threshold of 0.6, the recognition result is considered correct.  Figure 12 is the change curve of Loss with the number of iteration epochs during the training process of HE-Yolo. It can be seen that the Loss decreases rapidly at the beginning of the iteration, and it is stable between 3 and 4 after 65 iteration epochs.

### 3.2. The Evaluation Parameters

The precision rate *P*, the recall rate *R*, the average precision AP and the mean average precision mAP are selected as the parameters to evaluate the recognition performance of HE-Yolo. They are calculated as follows:

(6) $$\begin{array}{c} R=\frac{\text{TP}}{\text{TP}+\text{FN}}\times 100\%,\\ P=\frac{\text{TP}}{\text{TP}+\text{FP}}\times 100\%,\\ \text{AP}=\int_{0}^{1}\text{PRd}r,\\ \text{mAP}=\frac{1}{N}\sum_{N_{i}\in N}{\text{AP}}_{N_{i}}, \end{array}$$

where TP is the number of samples correctly recognized by the model, FP is the number of samples that the model misjudges as positive but negative, FN is the number of samples that the model misjudges as negative but positive, *N* is the category number of the pig-posture behaviors, *N*_*i*_ is the *i* th category and *i* ∈ [1,4], AP is the area of the P-R curve.

### 3.3. Selecting the Optimal Model

A total of 436 verification set images were used in 100 test stages, and the optimal model for all stages was selected. First of all, it is necessary to determine the priority of all evaluation parameters. The priority of evaluation parameters from small to large is *R*, *P,* and mAP. During the training process, the change curves of evaluation parameters with the number of iteration epochs are shown in Figure 13.

It can be seen from Figure 13 that the evaluation parameters grow fast in the first 70 epochs, and they are stable in the last 30 epochs. The mAP reaches the maximum value of 97.43% when the epoch is 96, and *P* reaches the maximum value of 96.79% when the epoch is 94. *R* reaches the maximum value of 97.64% when the epoch is 89. Therefore, HE-Yolo after 96 iteration epochs is selected as the optimal model to recognize the pig-posture behaviors.

### 3.4. Experimental Results and Analysis

#### 3.4.1. Analysis on the Recognition Results of HE-Yolo

Remove the SAM block in DAB to build the CA-Yolo, and remove the CAM block in DAB to build the SA-Yolo. The SSD [29] uses VGG16 as the backbone network, and the faster R–CNN uses the region generation network to replace the selective search in the fast R–CNN. Six models including HE-Yolo, CA-Yolo, SA-Yolo, Yolo v3, SSD and faster R–CNN are used to recognize four kinds of pig-posture behaviors, and the recognition results are listed in Table 2.

From Table 2 it can be known that:

1. Compared with Yolo v3, the AP values of HE-Yolo, CA-Yolo, and SA-Yolo for four postures are increased by 0.63%∼1.39%, 0.24%∼2.33%, 0.07%∼5.68%, and 0.48%∼4.04%, respectively, and the mAP values of three models are increased by 1.73%∼5.61%. That is, the introduction of an attention mechanism can improve the AP value of the model. The mAP value of SA-Yolo is higher than that of CA-Yolo, which shows that the spatial attention mechanism has an important influence on the recognition performance of the detection model. The AP values of a single category and the overall mAP value of HE-Yolo are higher than that of CA-Yolo and SA-Yolo, which shows that DAM can weaken the influence of noise on the recognition result of the detection model.
2. The AP values of HE-Yolo are higher than that of SSD and faster R–CNN, and its map value is also increased by 4.64% and 0.57%, respectively. Compared with Yolo v3, the single-frame recognition time of HE-Yolo increases by 0.007 s, but its map value increases by 5.61%. It can be seen from Table 2 that the mAP value of HE-Yolo is slightly higher than that of faster R–CNN, and from Table 3 it can be seen that the single-frame recognition time of HE-Yolo is reduced by 0.13 s.

Therefore, HE-Yolo has high recognition accuracy and fast recognition speed, which shows that HE-Yolo has strong mobility, and it can fully meet the real-time recognition requirement for the pig-posture behaviors.

#### 3.4.2. Recognizing the Images with Foreign Body Occlusion and Pig Adhesion

When the foreign body occlusion and pig adhesion are serious, the model is difficult to recognize the pig-posture behaviors.  Figure 14 shows the recognition results of HE-Yolo on the pig images with different degrees of foreign body occlusion and pig adhesion. Among them, there is partial foreign body occlusion and pig adhesion in Figures 14(a)∼14(b), and HE-Yolo can successfully recognize the pig-posture behaviors. There is serious foreign body occlusion and pig adhesion in Figure 14(c), and HE-Yolo cannot successfully recognize the pig-posture behaviors.

A total of 280 images with foreign body occlusion and pig adhesion are selected as the testing set, and the mAP value is used as the evaluation parameter. Four models including HE-Yolo, Yolo v3, SSD, and faster R–CNN are tested, and the experimental results are listed in Table 4.

It can be seen from Table 4 that the mAP value of HE-Yolo is 4.04%, 4.94%, and 1.76% higher than that of Yolo v3, SSD, and fast R–CNN, respectively. According to the actual observation and the recognition results, when HE-Yolo simultaneously extracts the feature information of three areas of the pig-limb, pig-abdomen, and pig-trunk, and the area covered by foreign body and pig adhesion is less than 25%, then HE-Yolo can effectively recognize the pig-posture behaviors.

#### 3.4.3. Analyzing the Influence of Lighting Condition on the Recognition Results

The images in the test set are divided into bright and dark according to the lighting conditions. Four models including HE-Yolo, Yolo v3, SSD, and faster R–CNN are used for the experiments, and the experimental results are listed in Table 5. It can be seen from Table 5 that the mAP values of HE-Yolo are the highest and its mAP values is only 1.24% different in two lighting conditions, which shows that HE-Yolo has good recognition performance under different lighting conditions.

The light varies greatly in the enclosure environment. To further test the robustness of HE-Yolo to the luminance of light, the RGB image is converted into an HSV image [30], and the luminance coefficient *α* of 10 gradients is set and *α* ∈ {0.5, 0.6, 0.7 … 1.5}. 10 luminance coefficients are multiplied by the luminance *V*, respectively, and then converted into RGB images to obtain the testing set with 10 different luminances. The experimental results of four models are shown in Figure 15.

It can be seen from Figure 15 that the stability of the mAP value of HE-Yolo is significantly better than that of other models, and the mAP values under 10 luminance conditions are higher than those of other models, which shows that HE-Yolo has stronger generalization ability and better robustness to the luminance of light, so it can meet the real-time recognition requirement of day and night alternation during the breeding process.

HE-Yolo is compared with other methods [3, 7, 12], and the mAP value, the training convergence epoch, and the single-frame recognition time are tested, respectively. The comparison results are listed in Table 6.

It can be seen from Table 6 that the mAP value of HE-Yolo is higher than that of other methods, and it converges after 65 iteration epochs, which shows that HE-Yolo needs lower hardware and less computation time, and its recognition speed is slightly lower than that of reference [7], but it can fully meet the real-time recognition.

## 4. Conclusion

In this study, HE-Yolo is built for real-time recognition of the pig-posture behaviors in the enclosure environment. HE-Yolo further optimizes the Yolo v3 model in structure, ensures the recognition effect and further reduces the computational complexity, and makes the new model more capable of focusing on effective features by constructing a multiple attention mechanism. The experimental results show that HE-Yolo has better accuracy and anti-interference ability than other models in a complex environment and provides a reliable research method for pig detection. The experiment results are summarized as follows:

The anchor boxes of Yolo v3 are optimized and clustered by the K-means algorithm. The depthwise separable convolution and h-switch activation function are introduced into Darknet-53 to build DBH, and C-Res unit with reverse inverse residual structure is designed to build Darknet-A feature extraction network to avoid network gradient explosion and ensure the integrity of image feature information.

According to the contribution of the feature information of different areas in the feature image, the spatial attention mechanism, and the channel attention mechanism are integrated to construct DAM, and the average pooling, the maximum pooling, the asymmetric convolution, 1 × 1 pointwise convolution and 3 × 3 depthwise convolutions together to form the Incep-abate module. DAM and the Incep-abate module are further combined to form DAB to reduce the computational complexity. DAB is spliced with the feature pyramid structure of Yolo v3 to make the model focus more on effective feature information, and HE-Yolo is finally built by Darknet-A and DAB.

Compared with Yolo v3, the mAP values of HE-Yolo, CA-Yolo, and SA-Yolo are increased by 5.61%, 1.73%, and 3.70%, respectively, which shows that the introduction of the attention mechanism can improve the extraction effect of effective features of the pig images. Among them, the mAP value of SA-Yolo is 1.97% higher than that of CA-Yolo, which shows that the spatial attention mechanism has an important influence on the recognition performance of the model.

The single-frame recognition time of HE-Yolo is 0.045 s, and its image recognition performance for foreign body occlusion and pig adhesion is good. The mAP value of HE-Yolo is 4.04%, 5.04% and 1.76% higher than that of Yolo v3, SSD, and faster R–CNN, and the mAP value of HE-Yolo is also higher than that of other models under different lighting conditions. Compared with other methods [3, 5, 7], HE-Yolo has high recognition accuracy and fast recognition speed under the condition of low hardware.

To sum up, the Yolo model designed in this paper has stronger generalization ability, can meet the real-time detection requirements of pig posture and behavior in the actual captive environment, has higher recognition accuracy and speed than other models, and has good robustness. Of course, HE-Yolo will be further optimized to improve its recognition performance and accurately track the pig-posture behaviors of individuals. In the next study, it cannot be limited to the abovementioned four posture behaviors, and the image data can be expanded for other types of pig-posture behavior or even be extended to other livestock.

## Figures and Tables

**Figure 1:** The image data after expansion.

**Figure 2:** The process of labeled images.

**Figure 3:** The structure of DPH unit.

**Figure 4:** The *h*-switch activation function.

**Figure 5:** The structure of C-Res unit.

**Figure 6:** The structure of SAM module.

**Figure 7:** The structure of CAM module.

**Figure 8:** The structure of DAM module.

**Figure 9:** Visualization of DAM feature extraction of pigs.

**Figure 10:** The structure of the Incep-abate module.

**Figure 11:** The structure of HE-Yolo.

**Figure 12:** The change curve of Loss with the number of iterations.

**Figure 13:** The change curves of *P*, *R,* and mAP.

**Figure 14:** The recognition results of HE-Yolo for different degrees of foreign body occlusion and pig adhesion. (a) Mild. (b) Medium. (c) Severe.

**Figure 15:** The recognition results of different models.

**Table 1:** The anchor box size and the corresponding output feature map after K-means clustering.

Size	13 × 13	26 × 26	52 × 52
Anchor box	(171 × 142), (168 × 114), (257 × 283)	(86 × 145), (105 × 70), (122 × 106)	(46 × 50), (72 × 93), (80 × 49)
Receptive field	Big	Middle	Small

**Table 2:** The recognition results of the pig-posture behaviors of the test set.

Model	AP (%)				mAP (%)
	Standing	Sitting	Prone	Sidling	
HE-Yolo	99.25	98.41	94.43	97.63	97.43
Yolo v3	97.86	96.08	88.75	93.59	91.82
CA-Yolo	98.49	96.32	88.82	94.07	93.55
SA-Yolo	98.96	96.68	91.01	95.43	95.52
SSD	97.55	94.39	86.32	92.86	92.78
Faster R–CNN	98.63	97.74	93.82	97.25	96.86

**Table 3:** Comparison of the single-frame recognition time.

Model	The single-frame recognition time (s)
HE-Yolo	0.045
Yolo v3	0.038
SSD	0.051
Faster R–CNN	0.175

**Table 4:** Recognition results of different models for foreign body occlusion and pig adhesion.

Model	HE-Yolo	Yolo v3	SSD	Faster R–CNN
mAP (%)	85.72	81.68	80.78	83.96

**Table 5:** The mAP values (%) of each model under different lighting conditions.

Type	Bright	Dark
Model		
HE-Yolo	98.12	96.88
Yolo v3	93.76	90.36
SSD	93.41	91.45
Faster R–CNN	97.21	95.53

**Table 6:** The comparison results of different methods.

Model	HE-Yolo	Literature [3]	Literature [7]	Literature [12]
mAP (%)	97.43	97.17	96.33	96.86
The training convergence epoch	65	74	86	58
The single-frame recognition time (s)	0.045	0.075	0.028	0.175

## Data Availability

The data used to support the findings of this study are available from the corresponding author upon request.
